# Synchronous Colorectal Liver Metastases considering Infectious Complications: Simultaneous or Delayed Surgery?

**DOI:** 10.1155/2022/5268554

**Published:** 2022-10-11

**Authors:** Lijun Huang, Xiao Tang, Jiafeng Fang, Zongheng Zheng, Hongbo Wei

**Affiliations:** Department of Gastrointestinal Surgery, The Third Affiliated Hospital of Sun Yat-sen University, Guangzhou 510630, Guangdong Province, China

## Abstract

**Background:**

Simultaneous or delayed surgery for synchronous colorectal liver metastases is performed in the clinic; which method is better is still up for debate. In particular, infectious complications are rarely compared. This study aims to investigate the differences between simultaneous and delayed surgery for synchronous colorectal liver metastases by comparing infectious complications and prognosis.

**Methods:**

Firstly, the patients' information from a single institution's database was retrospectively analyzed. Then the patients were divided into a simultaneous group and a delayed group according to synchronous colorectal liver metastases. Analyzing the postoperative complications within 30 days, the progression-free survival, and the overall survival in the two groups.

**Results:**

The simultaneous group had a higher neo-adjuvant chemotherapy rate (42.0% VS. 16.0% in the delayed group, *P* < 0.05) and laparoscopic surgery rate (89.8% VS. 72.0% in the delayed group, *P* < 0.05) than the delayed group. Moreover, the simultaneous group had a higher liver-related infection rate (17.0 VS. 0.0% in the delayed group, *P* < 0.05).

**Conclusion:**

Although there was no difference in survival rate between delayed and simultaneous surgeries, the delayed surgery have fewer liver-related infections compared with the simultaneous surgery in synchronous colorectal liver metastases patients. Delayed surgery could be a better treatment method for synchronous colorectal liver metastases patients.

## 1. Introduction

Colorectal cancer (CRC) is the third most frequent cancer disease, which claims more than 880,000 lives each year worldwide. It has been a major public health concern in the world [1–3]. Nearly 50% of CRC patients develop liver metastases, and at the time of initial diagnosis, 15% to 25% of CRC patients have synchronous liver metastases (SLM) [4]. Surgery containing resection or ablation of the liver metastasis is the curative way of dealing with the SLM [5]. A thorough resection of liver metastasis would improve survival and be associated with a 5-year survival rate of up to 40% [6–8]. However, the timing of the operation remains a matter of debate. Resection of synchronous colorectal liver metastasis can be performed via simultaneous surgery or delayed surgery. Simultaneous surgery means simultaneous resection on the same operative day. Delayed surgery indicates the two surgeries are carried out on separate operative days with a period of recovery. Compared with simultaneous surgery, delayed surgery is a traditional choice and focuses on the resection of the primary tumor first, followed by subsequent resection of the liver metastases in 3–6 months [9]. However, it is often thought that simultaneous surgery may avoid delayed removal of metastatic disease and reduce the risk of cancer spreading further [10]. However, it may lead to more surgical morbidity, especially in complex colorectal or liver resection, and should be considered [11].

Some retrospective and prospective studies reported that it was safe or not to treat liver metastasis along with primary cancer simultaneously. Compared with delayed liver surgery following resection of colorectal cancer, the simultaneous approach may have clear advantages in the hospital stay interval, the operation time, and most of all, avoiding another surgery [4, 12]. However, some studies report much higher mortality and severe complication rate in the simultaneous procedure [13, 14]. Therefore, the choice between simultaneous or delayed resection of the colorectal and liver remains controversial.

So far, most studies have compared the safety of the two methods in terms of postoperative complications. However, few studies pay close attention to infectious complications. As a common complication, perioperative infection not only influences the safety but also the long-term survival of the patients [5, 15]. Considering the complications of infection, more studies are needed on simultaneous and delayed surgery with simultaneous colorectal liver metastases. In our institution, the simultaneous way was well accepted, while the delayed way was chosen in a few cases, especially for some complex cases. It seems that the simultaneous surgery would lead to more infectious complications. Therefore, we conducted this retrospective study to compare the safety and prognosis of simultaneous surgery and delayed surgery. We aimed to investigate the differences between simultaneous and delayed surgery for synchronous colorectal liver metastases by comparing infectious complications and prognosis.

## 2. Materials and Methods

### 2.1. Samples Collection and Design

Colon cancer with liver metastasis patients who underwent liver resection from July 2011 to November 2020 in the Third Affiliated Hospital of Sun Yat-sen University was included.

#### 2.1.1. Inclusion Criteria

Age ≥18; histologically confirmed adenocarcinoma of the primary tumor; liver metastases found at the same time; no extrahepatic metastases; tumor R0 removing after the surgical treatments.

#### 2.1.2. Exclusion Criteria

Non-R0 resection of the hepatic lesions; hepatic lesions confirmed nonmetastases after surgery; extrahepatic metastases were found during the surgical interval of the delayed way.

The sample screening scheme was shown in Figure 1. Firstly, colorectal cancer patients with primary tumors and liver surgery (142 patients) were collected. After excluding repeated patients, patients with the nonmetastatic hepatic lesion, and patients with non-R0 resection, 113 patients were selected and divided into two groups: simultaneous group (*n* = 88) and delayed group (*n* = 25). The simultaneous group also called the synchronous group and defined as curative treatment of SLM, either with resection, radiofrequency ablation (RFA), or microwave ablation (MWA), was performed in one operation with resection of the primary tumor. While the delayed group was defined as curatively resecting the primary tumor first, followed by treatment of SLM a few months later. Examined variables including baseline clinic pathological data, operative factors, perioperative elements, infectious outcomes, and prognostic outcomes were collected by reviewing the hospital's archiving system or by contacting the patients and their treating doctors.

### 2.2. Data Definition and Management

For the delayed group, the bleeding volume and operation time in the separated surgery were added together to compare with the synchronous group. The overall survival (OS) time was defined as the time from the resection of the primary tumor to the death of the patient or the end point of follow up. The progression-free survival (PFS) time was defined as the time from the resection of the primary tumor to the progression of cancer or the end point of follow up. Complications were based on a standardized grading scale and the Clavien-Dindo classification of surgical complications [16]. This study was approved by the Ethics Committee of the Third Affiliated Hospital, Sun Yat-Sen University. The ethics number was [2022]02-031-01.

### 2.3. Statistical Analysis

Statistical analysis was performed using SPSS 21.0 (IBM SPSS Statistics 21.0). Continuous variables were expressed as mean ± standard deviation (SD), and any significant differences between the two groups were assessed by Student's *t*-test. Categorical variables were assessed by the chi-square test. Progression-free survival and overall survival were calculated using the Kaplan-Meier method, and differences in survival were estimated using the generalized log-rank test. In all analyses, *P* < 0.05 was considered to indicate statistical significance.

## 3. Results

### 3.1. Samples Screening and Analysis

As shown in Figure 1, data from these 113 patients were used to do the analyses. The endpoint of follow up was February 23, 2022. The median follow up time was 38 months (16–121 months). No one dropped off. To end, 40 patients died, and the overall survival rate was 64.6%.

The preoperative characteristics of the two groups were shown in Table 1. Totally, there were 79 males and 34 females; and the median age was 60.0 ± 12.8 years (age range 20–84 years). There was a similar distribution in gender, age, BMI, intestinal obstruction, abdominal infection, history of abdominal surgery, diabetes, cardiovascular disease, pulmonary disease, hepatic disease, smoking, alcohol abuse, site of the primary tumor, size of the primary tumor, differentiation, number of liver metastases, biggest size of liver metastases, location of liver metastases, parenteral nutrition, oral antibiotics preparation, and ASA score. While the synchronous group had fewer red blood cell transfusion rate compared with the delayed group (3.4% VS. 20.0%, *P*=0.004) and a higher neo-adjuvant chemotherapy rate (42.0% VS. 16.0%, *P*=0.017).

### 3.2. Comparison of Intraoperative Characteristics

As for the intro-operative characteristics (shown in Table 2), there are no differences in the right colectomy rate, stoma rate, and red blood cell transfusion rate. The difference between surgical way for liver lesions and combined organ resection among them was not significant (*P* > 0.05). They had similar bleeding volume and operation time, but the delayed group had a lower laparoscopic surgery rate for the primary tumor compared with the simultaneous group (72.0% VS. 89.8%, *P*=0.024).

### 3.3. Comparison of Postoperative Characteristics

As for the post operative characteristics, the comparison of Management, Pathology, and Clinical Risk Score (CRS) was operated on (Table 3). Moreover, the CRS, as a clinical score, is usually used to assess the risk of recurrence of colorectal cancer liver metastases, and 3–5 is divided into high risk of recurrence.

There was no perioperative death or severe liver failure. For the cases with complications, the total number was 37, and the hospital stay after surgery ranged from 10 to 107 days while the median was 14 days. Meanwhile, Table 4 showed that the simultaneous group had a higher liver-related infection rate (17.0 VS. 0.0% in the delayed group, *P*=0.027), but there was no difference in other complications between groups.

### 3.4. Comparison Analysis of PFS and OS between Groups

The PFS and OS rate trends were similar in both groups, which was shown in Figure 2. The 1-year, 3-year, and 5-year PFS rate was 54.5%, 37.0%, and 32.8% in the simultaneous group, while 48.0%, 8.9%, and 8.9% in the delayed group. As for OS rate, 96.6%, 64.8% and 55.5% in the simultaneous group and 96.0%, 70.3% and 58.7% in the delayed group, respectively.

## 4. Discussion

Surgical site infections, especially intro-abdominal infections, like liver abscesses and anastomotic leakage, can influence the safety and long-term survival of colorectal cancer patients with synchronous liver metastases after surgery [5, 15, 17, 18]. We firstly focused on the infectious complications after surgical treatments of CRC with SLM and found that the simultaneous group had a higher infection rate. These results suggested that surgeons should pay more attention to the liver-related infection when doing the synchronous procedure, not just the total surgical site infection rate. Doughtie et al. reported similar results [19]. They compared the infectious complications in combined colon resection and ablation of colorectal liver metastases and found that high-grade (grade, III to V) complications and liver-specific complications were significantly increased in the combined ablation group. In 2020, a meta-analysis study reported the overall morbidity rate in the simultaneous resection group was 39.2%, compared to 32.8% in the staged resection group, with a pooled number of 7639 patients. No significant difference was found (OR 1.04; 95% CI 0.89–1.22; *P*==0.63) [4]. The authors also gave data that compared anastomotic leaks, bile leaks, intra-abdominal abscesses, and subphrenic abscesses. The complication rates of the simultaneous resection group were all higher except for bile leak, but with no significant difference [4]. They did not compare the overall intro-abdominal infection rate. Another meta-analysis study containing 5300 patients in 2018 also confirmed that no statistically significant differences were found in safety and efficacy between the simultaneous and delayed hepatectomy cohorts, but the shorter length of hospital stay in the simultaneous group [20]. In 2021, a single prospective randomized controlled study was designed as a multi-center study with aimed at 222 enrolled patients. However, the enrollment was stopped at Number 85 due to no evidence of a difference in major complications between groups, and the potential of bad prognosis in the staged group [12]. When we went through the data again, the abdominal infection rate was 33.3% (13/39) in simultaneous resection and 13.0% (6/45) in delayed resection (*P* < 0.05). All these results suggested the safety of simultaneous colorectal and hepatic resection was unclear, and no study discussed the infectious complications alone. Our retrospective data showed that there might be more infections in simultaneous resection, suggesting that safety should be judged again.

It is still controversial whether synchronous colorectal cancer liver metastases (SLM) should be resected simultaneously with primary cancer or should be delayed. Firstly, both two procedures have their advantages and disadvantage. From the perspective of safety, the number of operations and anesthesia can be saved during the same period of surgery. Moreover, Gavriilidis et al. have reported that the hospital stay was significantly reduced during the same period of surgery [20]; However, a single operation may lead to a large wound area, much more operation time, and a high complication rate. Jessica Bogach et al. have even found in a retrospective cohort study that the 90-day postoperative mortality was higher[14], and the risk of each operation in a staged way might be low, but the interval between operations increased the number of chemotherapy, and might also increase the incidence of complications [21]. However, there was also some literature indicating that chemotherapy did not increase perioperative complications [22].

Furthermore, in terms of long-term prognosis, the preliminary results of a French multi-center randomized controlled study have shown that the staged group may have poor overall survival [5]. The main reason was that the disease progression of 8 cases in the staging group led to the termination of the experiment. This indicated that the study design was not perfect, and the oncology safety of the enrolled patients was not much enough considered. Thus, the results are not convincing. Bogach et al. have reported that simultaneous surgery may shorten the median overall survival (40 months, 95%CI 35–46 vs. 78 months, 95%CI 59–86) from a large retrospective cohort study [14]. Some recent reports have shown that PFS and OS are not significantly different, but the selection bias is obvious [4, 20]. Therefore, the pros and cons of these two surgical methods in terms of long-term survival are currently uncertain. Finally, it is still inconsistent about the definition of simultaneous liver metastasis of colorectal cancer in the published literature, including simultaneous discovery, and 3, 6, or 12 months separated, also cannot be homogenized [14]. Here are the results showing that based on the initial assessment of radically resectable concurrent liver metastases of colorectal cancer as the research object, the PFS and OS of concurrent surgery are equivalent to staged surgery. However, it may increase post-operative perihepatic infectious complications, which is similar to the conclusions of the published paper. The pros and cons of these two surgical methods still need to be clarified by high-quality research.

Nowadays, both surgical methods have been used in clinics. Our institution's experience was that, first, the surgical plan selection of the simultaneous or staged resection mainly depends on the evaluation of the liver surgeon. Second, because of the diverse surgical methods (TaTME and other surgical methods) for middle and lower rectal cancer [23], the operation is complicated and difficult, the complication rate of anastomotic leakage has significantly increased [24, 25], and the same period surgery should be avoided as much as possible. Therefore, when designing RCT studies, we should not include middle and low rectal cancer, and try to exclude the cases that cannot be controlled by systemic therapy, so as to avoid the case of prospective RCT in France, where the tumors of 8 staging cases have progressed to unresectable tumors. The study was terminated in advance with the conclusion that the prognosis of staged resection was poor [12]. From the meta-analysis and large population cohort studies [4, 14, 20], when the condition of the patients is good and liver and rectal lesion resection is relatively simple and safe, simultaneous surgery could avoid the problems caused by multiple operations. Further, the surgical safety and long-term prognosis are not weaker than staged surgery. Therefore, we speculated that both simultaneous and staged surgery have their advantages, but more research is needed to clarify the respective surgical indications. It may be a more meaningful direction to start from infection-related complications.

Due to the limitations of retrospective research, case selection may be biased; furthermore, the period is large, and the choice of treatment methods may be different. However, the results of our study still have certain guiding significance for the selection of surgical methods for this type of patient.

## 5. Conclusions

Delayed surgery for synchronous colorectal liver metastases may have fewer infectious complications, especially hepatic infections, than the simultaneous way with no different survival rate. High-quality prospective studies are still needed to detect which way is better or to set up the surgical indications for simultaneous colorectal and hepatic resection of colorectal cancer with synchronous liver metastases. And we should pay more attention to the hepatic infection rate in the following studies to confirm the benefit of the delayed way.

## Figures and Tables

**Figure 1:** Sample screening scheme diagram.

**Figure 2:** Comparison of the PFS (a) and OS, (b) between groups.

**Table 1:** Group information and characteristics of two groups.

Characteristics	Simultaneous group	Delayed group	*P* Value
	*n* = 88	*n* = 25	
Gender (male/female)	59/29	20/5	0.213
Mean age	60.1 ± 12.7	59.7 ± 13.4	0.908
BMI (kg/m2)	22.40 ± 3.25	22.76 ± 3.55	0.637
Intestinal obstruction (Y/N ^*∗*^)	13/75	7/18	0.126
Abdominal infection (Y/N)	1/87	1/24	0.338
History of abdominal surgery (Y/N)	12/76	3/22	0.831
Diabetes (Y/N)	15/73	5/20	0.733
Cardiovascular disease (Y/N)	28/60	5/20	0.251
Pulmonary disease (Y/N)	2/86	0/25	0.447
Hepatic disease (Y/N)	12/76	2/23	0.450
Smoking (Y/N)	17/71	3/22	0.398
Alcohol abuse (Y/N)	10/78	3/22	0.930
Site of primary tumor (right colon/left colon/rectum)	23/33/32	4/10/11	0.558
Size of the primary tumor (≤3 cm/>3 cm)	38/50	12/13	0.669
Differentiation (well or medial/poor)	79/9	22/3	0.800
Number of liver metastases	2.4 ± 1.8	2.4 ± 2.6	0.996
The biggest size of liver metastases (cm)	2.7 ± 1.6	2.2 ± 1.4	0.196
Location of liver metastases (right lobe/left lobe/both)	44/13/31	5/2/18	0.149
Red blood cell transfusion (Y/N)	3/85	5/20	0.004
Parenteral nutrition (Y/N)	7/81	3/22	0.994
Neo-adjuvant chemotherapy (Y/N)	37/51	4/21	0.017
Oral antibiotics preparation (Y/N)	28/60	9/16	0.694
ASA score (I, II/III, IV, V)	83/5	25/0	0.223

^*∗*^ Y/N is Yes/No.

**Table 2:** Comparison of intro-operative characteristics.

Characteristics	Simultaneous group	Delayed group	*P* value
	*n* = 88	*n* = 25	
Surgery for primary tumor (laparoscopic/open)	79/9	18/7	0.024
Right colectomy (Y/N)	23/65	4/21	0.294
Stoma (Y/N)	5/83	2/23	0.671
Surgery for liver lesions (ablation/resection/both)	61/22/5	22/3/0	0.147
Combined organ resection (Y/N)	1/87	0/25	0.592
Red blood cell transfusion (Y/N)	9/79	3/22	0.800
Bleeding volume (ml)	157.05 ± 353.51	78.40 ± 70.10	0.272
Operation time (min)	340.40 ± 97.66	324.08 ± 88.67	0.454

**Table 3:** Comparison of postoperative characteristics.

Characteristics		Simultaneous group *n* = 88	Delayed group *n* = 25	*P* value
Management	Time of preventive antibiotic use (POD^*∗*^)	4.76 ± 3.56	4.96 ± 2.68	0.797
	Time of abdominal drainage (POD)	4.55 ± 3.67	5.56 ± 7.67	0.356
	Postoperative hospital stay (POD)	14.07 ± 18.00	9.32 ± 7.44	0.053
	Postoperative chemotherapy	88/0	25/0	NA

Pathology	Tumor invasion (1–3/4)	24/64	3/22	0.114
	Lymph node (P/N^*∗∗*^)	59/29	20/5	0.213
	Vascular cancer thrombus (Y/N)	23/65	7/18	0.852
	Nerve invasion (Y/N)	18/70	9/16	0.108

CRS^*∗∗∗*^	1/2 VS. 3/4/5	13/33 VS. 39/3/0	2/13 VS. 10/0/0	0.455

*∗*POD, postoperation day; ^*∗∗*^P/N, positive/negative; ^*∗∗∗*^CRS, Clinical Risk Score.

**Table 4:** Occurred postoperative complications.

	Clavien-dindo grade^*∗*^	Simultaneous group	Delayed group	*P* value
		*n* = 88	*n* = 25	
Bleeding		8	1	0.278
	II/IIIa/IIIb/IVa/IVb	7/0/0/1/0	1/0/0/0/0	

Bowl obstruction		4	0	0.407
	II/IIIa/IIIb/IVa/IVb	4/0/0/0/0	0/0/0/0/0	

Liver-related infection		15	0	0.027
Bile leakage	II/IIIa/IIIb/IVa/IVb	0/1/0/0/0	0/0/0/0/0	
Abscess around liver	II/IIIa/IIIb/IVa/IVb	2/9/1/1/1	0/0/0/0/0	

Bowl-related infection		4	2	0.497
Anastomotic leakage	II/IIIa/IIIb/IVa/IVb	0/0/3/0/0	0/0/1/1/0	
Abscess around intestine	II/IIIa/IIIb/IVa/IVb	0/1/0/0/0	0/0/0/0/0	

Wound infection		7	1	0.333
	II/IIIa/IIIb/IVa/IVb	6/1/0/0/0	0/1/0/0/0	

Others^*∗∗*^		8	2	0.865
	II/IIIa/IIIb/IVa/IVb	6/1/0/1/0	1/0/0/0/1	
Total		32	5	0.124

^*∗*^Postoperative usage of analgesics and antiemetic is a routine treatment in our department. We cannot distinguish Grade 1 complications, so complications are defined as more than Grade 2. *∗∗*Other complications contain urinary tract infection, pulmonary infection, and catheter-related infection.

## Data Availability

The data used to support the findings of this study are available from the corresponding author upon request.
